The article "Severe Hypocalcemia due to Denosumab in Metastatic Prostate Cancer" was published in 2014. Journal: Case Rep Nephrol.

# Severe Hypocalcemia due to Denosumab in Metastatic Prostate Cancer

**DOI:** 10.1155/2014/565393

**Published:** 2014-06-26

**Authors:** Mohammed Muqeet Adnan, Usman Bhutta, Tanzeel Iqbal, Sufyan AbdulMujeeb, Lukas Haragsim, Syed Amer

**Affiliations:** ^1^Department of Internal Medicine, University of Oklahoma Health Sciences Center, Oklahoma City, OK 73117, USA; ^2^Department of Nephrology, University of Oklahoma Health Sciences Center, Oklahoma City, OK 73117, USA; ^3^University of Illinois at Chicago, Chicago, IL 60607, USA; ^4^Department of Internal Medicine, Mayo Clinic Hospital, Phoenix, AZ 85054, USA

## Abstract

Denosumab is a monoclonal antibody used for prevention of skeletal-related events (SREs) in patients with bone metastases from solid tumors. Hypocalcemia is a rare and dangerous side effect of the drug Denosumab. We present a case of a patient with metastatic prostate cancer who developed severe hypocalcemia after the administration of the drug. The patient's vitamin D levels were low when checked after administration of the drug, which likely predisposed him to the development of hypocalcemia. He was placed on high doses of oral and intravenous (IV) calcium and vitamin D without any appreciable response in the serum calcium level. His ionized calcium remained below 0.71 mmol/L despite very high doses of oral and IV calcium supplements. During the hospital course, he developed hydronephrosis from the spread of a tumor and did not want to undergo percutaneous nephrostomy tube placement; therefore, it was decided to dialyse him for acute renal failure and to correct his hypocalcemia. Checking calcium and vitamin D levels prior to the administration of Denosumab is vital in preventing hypocalcemia. If hypocalcemia is severe and not responsive to high doses of vitamin D, oral and IV calcium, then hemodialysis with a high calcium bath can correct this electrolyte abnormality.

## 1. Case Report

A 45-year-old gentleman with a three-year history of metastatic (bone, liver, and lymph nodes) prostate cancer and hypertension presented to the hospital with worsening leg swelling and hematuria. He had been treated with androgen deprivation therapy in the past, along with three doses of zoledronic acid for bone metastases. The bone pain was not controlled with the above regimen and it was decided to switch him to Denosumab. He received the dose approximately 13 days prior to hospitalization. Vitals at admission were significant for a blood pressure (BP) of 160/90 mmHg. Pertinent findings on physical examination were the presence of bilateral lower extremity edema and negative Chvostek and Trousseau's signs. The electrocardiogram showed a prolonged QT interval. Laboratory studies on admission revealed sodium of 135 mEq/L, potassium of 4.9 mEq/L, chloride of 105 mEq/L, bicarbonate of 23 mEq/L, blood urea nitrogen (BUN) of 22 mg/dL, creatinine of 1.34 mg/dL, glucose of 133 mg/dL, and calcium of 4.5 mg/dL, with albumin being 2.5 g/dL at admission. Phosphorus level was 6.1 mg/dL. The ionized calcium level at admission was 0.58 mmol/L. Laboratory studies done 13 days prior, when the drug was given, showed serum calcium of 8.4 mg/dL with an albumin of 2.9 g/dL. His vitamin D levels had not been checked prior to the administration of Denosumab. After admission to the hospital, his vitamin D 25-OH level was low at 12.1 ng/mL and vitamin D 1,25 dihydroxy level was high at 95.4 pg/mL. His initial PTH level was high at 440.7 pg/mL.

The article "Severe Hypocalcemia due to Denosumab in Metastatic Prostate Cancer" was published in 2014. Journal: Case Rep Nephrol.

He was started on 50,000 IU of ergocalciferol every 7 days, 2 mcg of calcitriol twice daily, and high doses of IV and oral calcium supplementation. Over the next 16 days, the patient received high doses of calcium carbonate; he was first started on 5 gm twice daily of calcium carbonate and 1337 mg of calcium acetate. Since the ionized calcium levels were consistently below 0.60 mmol/L, he was slowly increased to 10 gm twice daily of calcium carbonate and 3335 mg of calcium acetate thrice daily with meals. During the hospitalization, he received a total of 80 gm of IV calcium gluconate and 370 gm of oral calcium, but the highest ionized calcium level that could be achieved was 0.71 mmol/L. Figures 1 and 2 show the calcium and ionized calcium levels during the hospital while receiving oral and IV calcium supplementation.

He continued to have worsening lower-extremity edema, for which he was started on treatment with hydrochlorothiazide (HCTZ) to help with diuresis as well as with the hypocalcemia. His renal function kept worsening during his hospital stay and his creatinine reached 4.12 mg/dL. During workup for his renal failure, he was found to have hydronephrosis due to the spreading tumor. The options available were either placement of percutaneous nephrostomy tubes by interventional radiology to relieve the hydronephrosis and continued attempts at correction of his electrolytes via medical management or placement of a tunneled dialysis catheter and starting hemodialysis. After a discussion of the risks and benefits of each procedure and the overall prognosis of his condition, the patient opted for hemodialysis. Hemodialysis was initiated on the sixteenth day of hospitalization. He was dialysed daily for the next nine days with a high calcium bath along with two- to three-liter ultrafiltration daily to help get fluid off. His edema improved significantly, his serum calcium levels came above 8 mg/dL, and his ionized calcium stayed above 1 mmol/L without any IV supplementation; however, the oral supplementation with calcium acetate and 10 gm of calcium carbonate twice daily was continued. Due to the poor prognosis of the underlying disease, it was decided to send him home on hospice after arrangement of outpatient hemodialysis to prevent further hypocalcemia and maintain euvolemia. He died approximately three weeks later.

The article "Severe Hypocalcemia due to Denosumab in Metastatic Prostate Cancer" was published in 2014. Journal: Case Rep Nephrol.

## 2. Discussion

Denosumab is a fully human monoclonal antibody, administered subcutaneously, that inhibits osteoclast mediated bone resorption in bone metastases from solid tumors and multiple myeloma. It blocks the RANK ligand from activating the osteoclasts. Tumor cells secrete growth factors to stimulate osteoblasts to release RANK ligand. RANK ligand binds to RANK receptors on the osteoclasts and stimulates them to increase bone resorption. Denosumab blocks this action and hence a major part of calcium metabolism is blocked.

It has been approved by the US Food and Drug Administration (FDA) for use in postmenopausal women with risk of osteoporosis under the trade name Prolia and for the prevention of skeletal-related events in patients with bone metastases from solid tumors under the trade name XGEVA.

The recommended dose for XGEVA is 120 mg subcutaneously every four weeks, whereas for Prolia, it is 60 mg subcutaneous every six months.

The use of Denosumab is associated with a significantly increased risk of developing hypocalcemia [1, 2]. There have been very few case reports describing hypocalcemia to a great degree in patients who receive Denosumab [3]. One case report mentioned hypocalcemia in a dialysis patient after a single dose of Denosumab [3]. Patients are recommended to take 1000 mg oral calcium and 400 IU vitamin D daily in the insert for Prolia. The XGEVA insert recommends the administration of calcium and vitamin D as necessary to prevent hypocalcemia. None of the inserts recommend checking vitamin D levels prior to giving the drug or a certain vitamin D level below which the drug should not be administered.

We would like to emphasize the importance of checking and supplementing vitamin D levels prior to administration of this drug as well as checking serum calcium levels periodically after drug administration. Patients with low vitamin D levels can develop severe hypocalcemia that can be resistant to treatment. Patients might not always have symptoms of hypocalcemia until the serum calcium falls to dangerously low levels. Our patient did not have any of the classic symptoms of hypocalcemia (neuromuscular irritability, seizures, etc.) and presented to the hospital with worsening leg edema. The only manifestation of hypocalcemia that he had was a prolonged QT interval on electrocardiogram. Indeed, if he had not had leg swelling or hematuria, his hypocalcemia may not have been detected until he had a seizure or a fatal cardiac arrhythmia.

The article "Severe Hypocalcemia due to Denosumab in Metastatic Prostate Cancer" was published in 2014. Journal: Case Rep Nephrol.

There are cases reported of hypocalcemia after administration of denosumab, but very few cases showing such resistant hypocalcemia. Since our patient was on very high doses of oral and IV calcium, discharge was virtually impossible. We elected to start the patient on hemodialysis for two reasons: firstly, his worsening acute renal failure due to hydronephrosis, as he did not want to undergo percutaneous nephrostomy tubes placed; and secondly, his resistant hypocalcemia. Even if the patient did not have renal failure, we may have resorted to hemodialysis just to treat his hypocalcemia since all our options for medically managing the patient were getting exhausted without any real increase in the serum calcium level.

In patients who are already on dialysis, the hypocalcemia can be treated with a high calcium bath in addition to vitamin D supplement. However, in patients with normal renal function, hypocalcemia can usually be treated with a combination of oral and IV calcium along with activated vitamin D. In rare cases like these, hemodialysis with a high calcium bath may be an option.

In conclusion, we would recommend checking vitamin D 25 OH and serum calcium levels prior to starting treatment with Denosumab. Baseline phosphorus, albumin, and parathyroid hormone should also be checked prior to administration. If vitamin D levels are low, they should be supplemented prior to starting treatment. If treatment cannot be delayed to bring the vitamin D level within the normal range, then vitamin D supplement should be provided along with starting the drug. In either case, the serum calcium level should be monitored periodically to ensure that it does not fall below the normal range. Patients should be maintained on low doses of oral calcium and vitamin D daily while getting Denosumab to prevent hypocalcemia. It has been reported that the prophylactic administration of calcium 500 mg a day and vitamin D 400 IU daily can decrease the risk of hypocalcemia induced by Denosumab [2, 4]. Prolia is not expected to cause such severe hypocalcemia due to the low dose at six-month intervals. XGEVA, on the other hand, might be expected to cause more hypocalcemia since it is given at a higher dose and more frequently.

## Figures and Tables

**Figure 1:** Calcium levels while in the hospital remaining low despite ergocalciferol, calcitriol, and high doses of IV and oral calcium supplementation.

**Figure 2:** Ionized calcium levels during the hospital stay. Hemodialysis was initiated on day 16 due to worsening renal failure and persistent hypocalcemia.
